This article has been retracted.

# Frondoside A Suppressive Effects on Lung Cancer Survival, Tumor Growth, Angiogenesis, Invasion, and Metastasis

**DOI:** 10.1371/journal.pone.0053087

**Published:** 2013-01-08

**Authors:** Samir Attoub, Kholoud Arafat, An Gélaude, Mahmood Ahmed Al Sultan, Marc Bracke, Peter Collin, Takashi Takahashi, Thomas E. Adrian, Olivier De Wever

**Affiliations:** 1 Department of Pharmacology & Therapeutics, Faculty of Medicine & Health Sciences, U. A. E. University, Al-Ain, United Arab Emirates; 2 Laboratory of Experimental Cancer Research, University Hospital, Gent, Belgium; 3 Coastside Bio Resources, Stonington, Maine, United States of America; 4 Division of Molecular Carcinogenesis, Center for Neurological Diseases and Cancer, Nagoya University Graduate School of Medicine, Nagoya, Japan; 5 Department of Physiology, Faculty of Medicine & Health Sciences, U. A. E. University, Al-Ain, United Arab Emirates; H. Lee Moffitt Cancer Center & Research Institute, United States of America

## Abstract

A major challenge for oncologists and pharmacologists is to develop less toxic drugs that will improve the survival of lung cancer patients. Frondoside A is a triterpenoid glycoside isolated from the sea cucumber, *Cucumaria frondosa* and was shown to be a highly safe compound. We investigated the impact of Frondoside A on survival, migration and invasion *in vitro*, and on tumor growth, metastasis and angiogenesis *in vivo* alone and in combination with cisplatin. Frondoside A caused concentration-dependent reduction in viability of LNM35, A549, NCI-H460-Luc2, MDA-MB-435, MCF-7, and HepG2 over 24 hours through a caspase 3/7-dependent cell death pathway. The IC50 concentrations (producing half-maximal inhibition) at 24 h were between 1.7 and 2.5 µM of Frondoside A. In addition, Frondoside A induced a time- and concentration-dependent inhibition of cell migration, invasion and angiogenesis *in vitro*. Frondoside A (0.01 and 1 mg/kg/day i.p. for 25 days) significantly decreased the growth, the angiogenesis and lymph node metastasis of LNM35 tumor xenografts in athymic mice, without obvious toxic side-effects. Frondoside A (0.1–0.5 µM) also significantly prevented basal and bFGF induced angiogenesis in the CAM angiogenesis assay. Moreover, Frondoside A enhanced the inhibition of lung tumor growth induced by the chemotherapeutic agent cisplatin. These findings identify Frondoside A as a promising novel therapeutic agent for lung cancer.

## Introduction

Lung cancer is the most common form of cancer with one of the highest mortality rates in the world. Targeted therapies for selected subgroups of patients constitute a remarkable progress in the treatment of lung cancer. However, despite these advances, controversies remain, patients die, and a cure remains elusive [1]. Natural compounds are emerging as a new generation of anticancer agents with limited toxicity in cancer patients [2], [3]. They can have high value in tumors resistant to classical chemotherapies or resistant to tyrosine kinase inhibitors such as gefitinib

Sea cucumbers have been valued for hundreds of years in the Chinese diet as a food delicacy, as well as a medicine for a wide variety of diseases. In the United States and Canada, sea cucumber tissues are dried, pulverized and encapsulated as nutraceuticals for over-the-counter dietary health supplements, primarily directed at inflammatory conditions in humans and companion animals [4]. Frondoside A is a triterpenoid glycoside isolated from the Atlantic cucumber, *Cucumaria frondosa*. (See [5] for chemical structure). Recent studies demonstrate that low concentrations of Frondoside A inhibit the growth and induced apoptosis of human pancreatic, leukemia and breast cancer cells via caspase activation [6]–[8].

The chemotherapeutic agents currently in use for lung cancer are still unsatisfactory due to associated co-lateral toxicity and drug-induced resistance [9]–[11] which motivate our investigation of the impact of Frondoside A on human non-small cell lung cancer survival, migration and invasion *in vitro*, and on tumor growth, metastasis and angiogenesis *in vivo* alone and in combination with cisplatin.

## Materials and Methods

### Cell culture and reagents

Human lung cancer cells LNM35 (NSCLC) [12], A549 and NCI-H460-Luc2 (Caliper LifeSciences, US) were maintained in RPMI 1640 (Invitrogen, Paisley, UK), human melanoma MDA-MB-435, human mammary adenocarcinoma cells MCF-7, and human hepatoma cells HepG2 were maintained in DMEM (Invitrogen, Paisley, UK). All media were supplemented with antibiotics (penicillin 50 U/ml; streptomycin 50 µg/ml) (Invitrogen, Cergy Pontoise, France) and with 10% fetal bovine serum (FBS, Biowest, Nouaille, France). EndoGRO™ Human Umbilical Vein Endothelial Cells (HUVECs) (Millipore, Temecula, CA) were maintained in EndoGRO™^-^MV-VEGF Complete Media Kit (Millipore, Temecula, CA). Cisplatin was purchased from Sigma-Aldrich (Sigma-Aldrich, Saint-Quentin Fallavier, France). Frondoside A was purified from *Cucumaria frondosa*, harvested near Stonington, Maine and the purity (99.9%) confirmed by NMR as previously described [13], [14].

### Cellular viability

Cells were seeded at a density of 5,000 cells/well into 96-well plates. After 24 h, cells were treated for another 24 h with different concentrations of Frondoside A (0.01–5 µM), in triplicate. Control cultures were treated with 0.1% DMSO. The effect of Frondoside A on cell viability was determined using a CellTiter-Glo Luminescent Cell Viability assay (Promega Corporation, Madison, USA), based on quantification of ATP, which signals the presence of metabolically active cells. The luminescent signal was measured using the GLOMAX Luminometer system. Data were presented as proportional viability (%) by comparing the treated group with the untreated cells, the viability of which is assumed to be 100%.

### Caspase 3/7 activity

LNM35 cells were seeded at the density of 5,000 cells/well into 96-well plate and treated with Frondoside A (1–2.5 µM) for 2 and 24 h, in triplicate. Caspase-3/7 activity was measured using a luminescent Caspase-Glo 3/7 assay kit following the manufacturer's instructions (Promega Corporation, Madison, USA). Caspase reagent was added and the plate was mixed using an orbital shaker and incubated for 2.5 h at room temperature. Luminescence was measured using a GLOMAX Luminometer system.

### Wound healing motility assay

LNM35 cells were grown in six-well tissue culture dishes until confluence. Cultures were incubated for 10 min with Moscona buffer. A scrape was made through the confluent monolayer with a plastic pipette tip of 1 mm diameter. Afterwards, the dishes were washed twice and incubated at 37°C in fresh RPMI containing 10% fetal bovine serum in the presence or absence of the non-toxic concentrations of Frondoside A (0.1–0.5 µM). At the bottom side of each dish, two arbitrary places were marked where the width of the wound was measured with an inverted microscope (objective ×4) (Olympus 1X71, Japan). Motility was expressed as the average ± S.E.M of the difference between the measurements at time zero and the 6, 24 and 30 h time period considered.

### Matrigel invasion assay

The invasiveness of the lung cancer cells LNM35 treated with Frondoside A (0.1–1 µM) was tested using BD Matrigel Invasion Chamber (8-µm pore size; BD Biosciences, Le Pont de Claix, France) according to manufacturer's protocol. The PI3 kinase inhibitor LY294002 (20 µM) was used as a positive inhibitor of cellular invasion. Briefly, Cells (1×10^5^ cells in 0.5 mL of media and the indicated concentration of Frondoside A) were seeded into the upper chambers of the system, the bottom wells in the system were filled with RPMI supplemented with 10% fetal bovine serum as a chemo-attractant and then incubated at 37°C for 24 h. Non-penetrating cells were removed from the upper surface of the filter with a cotton swab. Cells that have migrated through the Matrigel were fixed with 4% formaldehyde, stained with DAPI and counted in 25 random fields under a microscope. The assay was carried out in duplicate and repeated three times for quantitative analysis.

### Chorioallantoic membrane (CAM) angiogenesis assay

This assay was performed as described previously [15], with some modifications. Briefly, fertilized eggs were incubated for 3 days at 37, 8°C with a humidity of 48%. On day 4, albumen was removed to detach the shell from the developing CAM and a window was made in the eggshell, exposing the CAM, and covered with a breathing film (suprasorb F®). The eggs were returned to the incubator until day 10, prior to application of the test compounds. Test compound and control compound (DMEM without 10% FBS) dissolved in DMEM without 10% FBS were poured onto separate sterile discs (12 mm diameter), which were allowed to dry under sterile conditions. A solution of cortisone acetate (125 µg/disc) was poured onto all discs to prevent an inflammatory response. Test discs probed with recombinant human bFGF (Peprotech) served as a control for angiogenesis stimulation. On each CAM, the disc containing control compound and the disc containing test compound were placed at a distance of 1 cm. The windows were covered and the eggs were incubated until day 14, before assessment of angiogenesis. Therefore, the eggs were flooded with 10% buffered formalin and the eggs were kept at room temperature for at least 20 minutes. The CAM, the area of the discs included, was placed in a petri dish with 10% buffered formalin. The plastic discs were removed and phase-contrast pictures of the area of the plastic discs were taken. The vascular index was measured as described previously [16]. Vascular intersections on a grid containing three concentric circles (6, 8 and 10 mm diameter with as center the center of the disc) were counted. The angiogenic index = *(t-c)/c*, with *t* the number of intersections in the area covered by the test disc and *c* the number of intersections in the area covered by the control disc in the same egg. The Mann-Whitney U-test was used for statistical analysis (p<0.05).

### Vascular tube formation assay

Assessment of *in vitro* capillary formation used Matrigel (Becton Dickinson, Le Pont de Claix, France). Matrigel is a squamous cell carcinoma basement membrane matrix composed primarily of collagen IV, laminin, entactin, and heparan sulfate proteoglycans. The Matrigel matrix was thawed, gently mixed to homogeneity using cooled pipettes, and diluted v/v with the EndoGRO™^-^MV-VEGF Complete Media Kit medium (Millipore, Temecula, CA, USA). Matrigel, 50 µl/well, supplemented with angiogenic peptides and other effectors was used to coat the wells of 96-well plates. The plate was then incubated for one hour at 37°C to allow the matrix solution to solidify prior to treatment. HUVECs (at a density of about 4×10^4^ cells/well and the indicated concentration of Frondoside A) were plated to each well and incubated for 8 h at 37°C in 0.1 mL of EndoGRO™^-^MV-VEGF Complete Media Kit medium (Millipore, Temecula, CA, USA). Then cells were photographed using an inverted phase contrast photomicroscope. The tubular network growth area was compared in control and inhibitor-treated Matrigel matrix. Tube formation was quantified by counting the number of tube-like structures formed in each well. The effect of Frondoside A on viability of the HUVEC was determined using a CellTiter-Glo Luminescent Cell Viability assay (Promega Corporation, Madison, USA), as previously described for the cancer cells.

### Tumor growth and metastasis assay

The animal experiments were performed in accordance with the protocol approved by the animal ethics committee and the Institutional Animal Care at the Faculty of Medicine & Health Sciences/UAE University. Six-week-old athymic NMRI female nude mice (nu/nu, Charles River, Germany) were housed in filtered-air laminar flow cabinets and handled under aseptic conditions. Procedures involving animals and their care were conducted in conformity with Institutional guidelines that are in compliance with Faculty of Medicine & Health Sciences, national and international laws and policies (EEC Council Directive 86/609, OJ L 358, 1, December 12, 1987; and NIH Guide for Care and Use of Laboratory Animals, NIH Publication No. 85-23, 1985). LNM35 cells (1×10^6^ cells in 200 µl PBS) were injected subcutaneously into the lateral flank of the nude mice. One week after inoculation, when tumors had reached the volume of approximately 150 mm^3^, animals (six in each group) were treated in the first protocol for 25 days with Frondoside A (0.01 and 1 mg/kg/day, ip) or carrier solution (control) in order to determine the effect of Frondoside A alone on tumor growth and metastasis. In the second protocol, animals were treated for only 10 days with the lowest dose of Frondoside A (0.01 mg/kg/day, ip), cisplatin (1 mg/kg/day, ip), or with combined Frondoside A and cisplatin treatment. Control animals were treated with carrier solution. Tumor dimensions and animal weights were measured every 3 days. Tumor volume (V) was calculated using the formula: V = 0.4×a×b^2^, with “a” being the length and “b” the width of the tumor. After sacrifice, the tumors and axillary lymph nodes were excised and weighed.

### Immuno-histochemical determination of CD31/platelet-endothelial cell adhesion molecule 1 (PECAM-1) for Microvessel Density

The effect of Frondoside A on angiogenesis was evaluated using CD31 immuno-staining. The tumor tissues were quickly frozen in isopentane at −130°C and stored at −70°C until further processing. Eight-µm frozen sections were fixed in acetone, and incubated overnight with a CD31 antibody (clone MEC13.3, 1∶100) (BD Pharmingen, San Jose, CA, USA). Slides were then washed three times in PBS and incubated with secondary antibody labeled with rhodamine (goat anti-rat 1∶100) for one hour at room temperature. The area occupied by CD31-positive microvessels and total tissue area per section were compared between treated and control mice. All analyses were performed in a blind fashion.

Results were expressed as means ± S.E.M. of the number of experiments. The difference between experimental and control values were assessed by ANOVA followed by Dunnett's post-hoc multiple comparison test. Tumor growth and metastasis studies were analyzed using the unpaired Student's t-test. P<0.05 indicate a significant difference.

## Results

### Effect of Frondoside A on cellular viability

As shown in **fig. 1**, Frondoside A concentrations (0.01–5 µM) caused a concentration-dependent decrease in cell viability of LNM35, A549, NCI-H460-Luc2, MDA-MB-435, MCF-7, and HepG2 cells over 24 hours. The IC50 concentrations (producing half-maximal inhibition) at 24 h were in the range of 1.7 and 2.5 µM Frondoside A for all cell lines.

**Figure 1:** Inhibition of cellular viability by Frondoside A. Exponentially growing LNM35 (**A**), A549 (**B**), NCI-H460-Luc2 (**C**), MDA-MB-435 (**D**), MCF-7 (**E**), and HepG2 (**F**) cells were treated with vehicle (0.1% DMSO) and the indicated concentrations of Frondoside A. Viable cells were assayed as described in Materials and Methods. All experiments were repeated at least three times. *Columns*, mean; *bars*, S.E.M. **Significantly different at P<0.01, ***Significantly different at P<0.001.

### Frondoside A induces caspase-3/7 activation

Caspase-3/7 activity is essential in apoptotic cell death pathways. The relative activity of caspases 3/7 was analyzed in LNM35 cells treated for 2 and 24 h with Frondoside A (1–2.5 µM), and normalized to the number of cells per well. As shown in **Fig. 2**, caspase 3/7 activity increased by 2.5- and 10.8-fold in LNM35 cells treated for 24 h with Frondoside A 1 and 2.5 µM respectively. Similar effect was observed after treatment with Frondoside A (1–2.5 µM) for 2 h (data not shown).

**Figure 2:** Induction of caspase-3/7 activity was analyzed in LNM35 cells treated for 24 h with Frondoside A (1–2.5 µM), normalized to the number of viable cells per well and expressed as fold induction compared with the control group. *Significantly different at P<0.05.

### Impact of Frondoside A on LNM35 xenografts

To confirm the pharmacological relevance of our *in vitro* data, the anticancer activity of Frondoside A was investigated *in vivo* in athymic mice inoculated with LNM35 lung cancer cells. The growth of the LNM35 human tumor xenografts was monitored every third or fourth day for 25 consecutive days after daily i.p. injection of 0.01 mg and 1 mg/kg of Frondoside A. Treatment with the lowest dose of Frondoside A (0.01 mg/kg/day) reduced the volume of the LNM35 xenografts by 41% (**Fig. 3A**). A similar difference was also found in tumor weight at the end of the experiment (2.1+/−0.3 g versus 4.5+/−0.8 g; *P<0.05*; **Fig. 3C**). Treatment with the highest dose (100 times more) of Frondoside A (1 mg/kg/day) reduces about 43.9% tumor volume of the LNM35 xenografts (**Fig. 3B**). Almost similar difference was found in tumor weight at the end of the experiment (3+/−0.5 g versus 4.5+/−0.8 g; **Fig. 3D**). This experiment clearly demonstrated that the lowest dose of Frondoside A (0.01 mg/kg/day) is optimal for the inhibition of tumor growth. There were no manifest undesirable effects of Frondoside A treatment on animal behaviour or body weight in either experiment (**Fig. 3E and 3F**). In addition, there were no visible abnormalities at necropsy, or any other obvious signs of toxicity as previously described by our team [**7**].

**Figure 3:** Frondoside A induces regression of established LNM35 xenografts. **A) & B**) Tumor volume of LNM35 xenografts inoculated subcutaneously in nude mice and treated with Frondoside A (0.01 and 1 mg/kg, intra-peritoneal injections, respectively) or control carrier solution alone, for a total of 25 days. Data points represent the mean ± S.E.M. of 6 mice per group. **C) & D**) Tumor weight obtained from the same control and treated nude mice. Data points represent the mean ± S.E.M. of 6 mice per group. *Columns*, mean; *bars*, S.E.M. **E) & F**) Body weight of these mice. Data points represent the mean ± S.E.M. of 6 mice per group. *Significantly different at P<0.05.

### Inhibition of angiogenesis by Frondoside A in the xenografted tumors and the CAM assay *in vivo* and in the capillary-like structures *in vitro*

Angiogenesis is an attractive target in cancer therapy not only because it supplies oxygen and nutrients for the survival of tumor cells but also provides the route for metastatic spread of these cancer cells. First, we demonstrate that in the proliferating areas at the periphery of the tumor, microvessel density (measured by CD31 staining) was significantly reduced by Frondoside A (0.01 mg/kg/day) (**Fig. 4, right panel**) in comparison with the control-treated tumors (**Fig. 4, left panel**). Next, we used the CAM assay involving the coordination and integration of multicellular responses during development of the chick embryo to confirm this potential anti-angiogenic effect of Frondoside A. As shown in **Fig. 5** **and** **6**, bFGF (2 µg/ml), stimulated 15% new vessel formation with angiogenic indices statistically different compared with the control DMEM medium. Frondoside A (100 and 500 nM) inhibited basal angiogenesis in a concentration-dependent manner with respectively 7% and 12% inhibition of angiogenic index compared to control (**Fig. 5** **and** **6**). The formation of new blood vessels induced by bFGF was also completely suppressed by Frondoside A (500 nM) (**Fig. 5** **and** **6**). Finally, to assess whether the anti-angiogenic effect of Frondoside A involves a direct interaction of the compound with endothelial cells, we conducted comparative studies on the formation of capillary-like structures *in vitro*, using HUVECs plated on Matrigel-coated plates. As shown in **Fig. 7A**, human endothelial cells have the ability to form capillary structures when seeded and cultured on top of Matrigel substrate. Control cells move from their initial uniform pattern of dispersed cell layers and associate to form a network of cell clusters connected by long, multicellular processes leading to the formation of tube-like structures. Addition of non-toxic concentrations of Frondoside A (0.01–1 µM) resulted in a marked inhibition of this spontaneous angiogenic phenotype (**Fig. 7A, and 7B**). Frondoside A induced inhibition of this spontaneous angiogenic phenotype occurred without significant reduction of cell viability (**Fig. 7C**). Taken together, these data confirm a strong anti-angiogenic potential of Frondoside A.

**Figure 4:** The anti-angiogenic activity of Frondoside A in the xenograft tumor: Immuno-histochemical staining of lung xenograft tumors for CD31 (microvessel density).

**Figure 5:** The anti-angiogenic activity of Frondoside A in the Chorioallantoic membrane (CAM) assay *in vivo*: CAM was treated with control (serum-free medium), 100 nM Frondoside A, 500 nM Frondoside A, 2 µg/mL bFGF, 2 µg/mL bFGF+500 nM Frondoside A and the vascularization of test discs was photographed.

**Figure 6:** Quantification of CAM angiogenesis assay: *Bars* indicate angiogenic indices (%) of CAM's probed with 2 µg/mL bFGF, 100 nM Frondoside A, 500 nM Frondoside A, 2 µg/mL bFGF+500 nM Frondoside A. Data represents mean ± SD (Mann-Whitney U-test, *: p<0.05, ***: p<0.01). In each experiment, six eggs were tested per condition.

**Figure 7:** Impact of Frondoside A on the formation of capillary-like structures by HUVECs *in vitro*. **A**) Patterns of angiogenesis induced by human umbilical vein endothelial cells (HUVEC) cultured on Matrigel matrix in 96-well plates in the absence or presence of the Frondoside A. **B**) Quantification of tubular morphogenesis induced in HUVEC cells cultured in the absence or presence of Frondoside A. Tube formation was determined by the length of tube-like structures containing connected cells. Data are mean ± S.E.M. from three separate experiments. Asterisks indicate that significantly different values were obtained in the presence of the indicated inhibitors vs. the corresponding control stimulation. ***Significantly different at P<0.001. **C**) HUVEC cells were treated with vehicle (0.1% DMSO) and the indicated concentrations of Frondoside A. Viable cells were assayed as described in Materials and Methods. All experiments were repeated at least three times. *Columns*, mean; *bars*, S.E.M.

### Frondoside A also impairs lung cancer cell migration and invasion *in vitro* and metastasis *in vivo*

Cancer progression is associated with the abrogation of normal controls that limit cell migration and invasion, eventually leading to metastasis. Lung cancer patients are at high risk of recurrence in the form of metastatic disease. Metastasis starts with cell migration in the primary tumor, leading to local tissue invasion and entry into lymph or blood vessels. The ability of Frondoside A to reduce cellular migration was investigated using a classic *in vitro* wound healing model. Frondoside A reduced cellular migration of LNM35 cells in a concentration- and time-dependent manner (**Fig. 8A**). Similarly, Frondoside A impaired the invasion of LNM35 cells in matrigel invasion assay (**Fig. 8B**). Frondoside A induced inhibition of cellular migration and matrigel invasion occurred without significant reduction of cell viability (**Fig. 1A**).

**Figure 8:** Frondoside A also impairs lung cancer cell migration and invasion *in vitro* and metastasis *in vivo*. **A**) Wounds were introduced in LNM35 confluent mono-layers cultured in the presence or absence (control) of Frondoside A (0.1–0.5 µM). The mean distance that cells travelled from the edge of the scraped area for 6, 24, and 30 h at 37°C was measured in a blinded fashion, using an inverted microscope (4× magnifications). Data are means ± S.E.M. of two independent experiments. **B**) LNM35 cells were incubated for 24 h in the presence or absence of Frondoside A (0.01–1 µM) and LY294002 (20 µM). Cells that invaded into Matrigel were scored as described in Materials and Methods. *Columns*, mean; bars, S.E.M. Lymph nodes metastasis weight of established human lung cancer xenografts treated with Frondoside A 0.01 mg/kg (**C**) and 1 mg/kg (**D**) every day for 25 days. *Columns*, mean; *bars*, S.E.M. *Significantly different at P<0.05, **Significantly different at P<0.01, ***Significantly different at P<0.001.

Next, we assessed the metastatic behavior of the human pulmonary cell line LNM35 by examining axillary lymph nodes. Histological examination of the lymph nodes in LNM35-bearing mice revealed the presence of LNM35 cells in all lymph nodes from both the control and Frondoside A treated mice (data not shown). In the control-treated group, the mean lymph nodes weight was 548.5+/−112.8 mg compared with 256+/−43.3 and 268.8+/−55.7 mg in the groups treated with Frondoside A 0.01 mg and 1 mg/kg/day, respectively (**Fig. 8C and 8D**).

### Frondoside A enhances the anticancer activity of cisplatin

As shown in **Fig. 9A**, daily administration of Frondoside A to nude mice reduced the growth of LNM35 human tumor xenografts by 40.3% at day 10. Inhibition of LNM35 tumor xenograft growth by Frondoside A was comparable with that produced by the DNA-damaging anticancer agent cisplatin (46.9%). Combined treatment of Frondoside A with cisplatin resulted in a remarkable potentiation (67.6%; *P<0.05*) of the cisplatin therapeutic effect (**Fig. 9A**). There were no manifest side effects of the combined treatment on animal behaviour or body weight (**Fig. 9B**).

**Figure 9:** Antitumor activity of Frondoside A alone or in combination with the anticancer drug, cisplatin, against human lung tumor xenografts in athymic nude mice. **A**) Frondoside A enhances cisplatin efficacy against NSCLC LNM35 cells growing as xenografts. **B**) Impact of Frondoside A and cisplatin alone or in combination on body weight. *Significantly different at P<0.05.

## Discussion

Despite advances in molecular biology of lung cancer, improved diagnosis, and even optimal target therapies, the current protocols for the treatment of lung cancer are still insufficient to produce striking clinical benefits and the cure of lung cancer patients remains unsuccessful. The current targeted therapy drugs develop resistance and they are very expensive and not available to the majority of lung cancer patients in the world. Many drugs have relatively low activity; few patients are cured, with a brief, if any, increase in survival [17]. The history of anti-cancer agents, such as paclitaxel, shows that the mechanism of action was identified several years after its clinical efficacy was demonstrated. Despite not knowing the drug's mechanism of action, we believe that the *in vitro* as well as the strong *in vivo* anti-cancer effects of Frondoside A should translate in the clinic to a new potent anti- lung cancer agent.

In the present study, we investigated the impact of Frondoside A on lung cancer cells progression. We showed that Frondoside A caused concentration-responsive (0.01–5 µM) decreases in viability of LNM35, A549, and NCI-H460-Luc2 cells over 24 hours through the caspase 3/7-dependent cell death pathway. The IC50 concentrations (producing half-maximal inhibition) at 24 h were between 1.7 and 2.5 µM Frondoside A. These results are consistent with previously published results that low concentration of Frondoside A inhibits the growth of human pancreatic cancer cells and induced apoptosis through caspase 9/3/7, increased bax, decreased bcl-2 and mcl-1, and arrested cell cycle and up-regulated p21 [8], induced apoptosis in human leukemia cells via caspase activation [6], and significantly decreases the viability of the estrogen receptor (ER)-negative MDA-MB-231 breast cancer cells by inducing apoptosis via the Caspase9-Caspase3/7 intrinsic pathway [7]. It has also been demonstrated that Frondanol A5, an impure extract of *Cucumaria frondosa* skin from which Frondoside A is originally derived, induced growth inhibition at S and G2-M phase with a decrease in Cdc25c and an increase in p21^WAF1/CIP1^ with significant apoptosis associated with H2AX phosphorylation and caspase-2 cleavage in the colon cancer-derived HCT116 cells [4]. A second paper also demonstrated that Frondanol-A5P, a polar precipitate sub-fraction of Frondanol-A5, inhibited proliferation and induced G2/M phase cell cycle arrest in two pancreatic cancer cells with decreased expression of cyclin A, cyclin B, and cdc25c [18]. This anticancer effect of Frondoside A is not tissue specific, and in this context we demonstrated that Frondoside A induced a concentration-dependent decrease in cell viability of the melanoma MDA-MB-435, the breast MCF-7, and the hepatoma HepG2 cells.

To assess the effects of Frondoside A on lung tumor development *in vivo*, LNM35 xenografts were made in immuno-suppressed mice. We demonstrated that intraperitoneal administration of Frondoside A caused a strong regression of established tumors. Maximum inhibition was obtained with the low dose of 0.01 mg/kg/day for 25 days. A 100 times higher dose gives similar effects indicating that increasing the dose will not improve the anti-cancer efficacy of Frondoside A. The cancer inhibitory effect of Frondoside A has been observed previously on AsPC-1 pancreatic and MDA-MB-231 xenografts in athymic mice [7], [8]. This anti-tumor effect of Frondoside A may be partly due to its immuno-stimulatory effect [13] and/or anti-angiogenic effect. In this study, we demonstrated for the first time, that Frondoside A is a strong anti-angiogenic agent. It reduces the microvessel density (measured by CD31 staining) in the xenografted tumor treated with Frondoside A and also significantly reverse basal and bFGF induced angiogenesis in the CAM angiogenesis assay. Similarly, Frondoside A completely suppressed capillary structure formation on Matrigel substratum by human endothelial cells.

Angiogenesis is an attractive target in cancer therapy not only because it supplies oxygen and nutrients for the survival of tumor cells but also provides the route for metastatic spread of these cancer cells. Cancer progression is associated with abrogation of the normal controls that limit cell migration and invasion, leading eventually to metastasis. As metastasis is the major cause of death in cancer patients, the development of new treatment regimens that reduce invasion and metastasis is highly important in cancer therapy. In this context, we demonstrated that Frondoside A induced a highly significant time- and concentration-dependent inhibition of cell migration, invasion *in vitro* and metastasis *in vivo*. These results are in agreement with our previous study showing that Frondoside A at concentrations that are not cytotoxic to the cells exerts a strong inhibitory effect on both the migratory and invasive properties of MDA-MB-231 breast cancer cells [7] and with another recent study demonstrating that Frondoside A inhibits breast cancer metastasis to the lungs [19].

Building on aforementioned results, and knowing from clinical trials that single agent treatments rarely result in clinical benefits to cancer patients, and that combination therapy are necessary for effective treatment of tumors, we investigated the therapeutic advantage of combination of cisplatin, (a first line treatment of lung cancer), with Frondoside A in nude mice bearing LNM35 xenografts. We found that Frondoside A enhances the inhibition of lung tumor growth induced by the chemotherapeutic agent cisplatin. These findings identify Frondoside A as a promising novel therapeutic agent for lung cancer and perhaps other cancers too.
